# Heartbeat Classification Based on Multifeature Combination and Stacking-DWKNN Algorithm

**DOI:** 10.1155/2021/8811837

**Published:** 2021-01-28

**Authors:** Shasha Ji, Runchuan Li, Shengya Shen, Bicao Li, Bing Zhou, Zongmin Wang

**Affiliations:** ^1^School of Information Engineering, Zhengzhou University, Zhengzhou 450000, China; ^2^Cooperative Innovation Center of Internet Healthcare, Zhengzhou University, Zhengzhou 450000, China; ^3^Zhengzhou University of Economics and Business, Zhengzhou Henan, Zhengzhou 450000, China; ^4^Zhongyuan University of Technology, Zhengzhou Henan, Zhengzhou 450000, China

## Abstract

Arrhythmia is one of the most common abnormal symptoms that can threaten human life. In order to distinguish arrhythmia more accurately, the classification strategy of the multifeature combination and Stacking-DWKNN algorithm is proposed in this paper. The method consists of four modules. In the preprocessing module, the signal is denoised and segmented. Then, multiple different features are extracted based on single heartbeat morphology, P length, QRS length, *T* length, PR interval, ST segment, QT interval, RR interval, *R* amplitude, and *T* amplitude. Subsequently, the features are combined and normalized, and the effect of different feature combinations on heartbeat classification is analyzed to select the optimal feature combination. Finally, the four types of normal and abnormal heartbeats were identified using the Stacking-DWKNN algorithm. This method is performed on the MIT-BIH arrhythmia database. The result shows a sensitivity of 89.42% and a positive predictive value of 94.90% of S-type beats and a sensitivity of 97.21% and a positive predictive value of 97.07% of V-type beats. The obtained average accuracy is 99.01%. Compared to other models with the same features, this method can improve accuracy and has a higher positive predictive value and sensitivity, which is important for clinical decision-making.

## 1. Introduction

Cardiovascular disease is one of the main diseases that endanger human health [1]. Arrhythmia is a common cardiovascular syndrome, and accurate identification of arrhythmia is an essential part of the prevention of cardiovascular diseases. Most arrhythmias are harmless, but some may immediately threaten people's lives. Early detection of arrhythmia can prolong life through proper treatment. The electrocardiogram (ECG) is a popular and mature diagnostic tool. It contains basic physiological information for analyzing cardiac function [2] and is the most basic method for the diagnosis of arrhythmia. Different classes of arrhythmias can be detected by analyzing the changes of ECG waveform, but it usually needs to be diagnosed at the onset of the disease. Some patients' symptoms appear infrequently. Traditional electrocardiogram may not capture the electrocardiogram at the time of onset. It is necessary to use dynamic ECG to record long-term cardiac electrical activities [3].

It may be time-consuming and impractical to rely on manual analysis of ECG signals. Moreover, due to the interference of noise and the diversity of ECG waveforms, arrhythmia is difficult to accurately diagnose and easy to be misdiagnosed. At the same time, relying on manual recognition of electrocardiograms often lacks real-time, which may delay the best time for patient treatment. The application of computer-aided intelligent diagnosis to the classification of arrhythmias can help doctors more accurately diagnose arrhythmias and reduce the workload of doctors. In the literature, numerous algorithms have been proposed to achieve an accurate result for the classification, mainly including deep learning-based approaches and feature extraction-based approaches.

Deep neural networks usually work in an end-to-end way, do not require manual feature extraction, and are widely used for ECG classification [4]. However, although they are good at learning feature representations and have produced very competitive performance in a wide range of applications, they cannot analyze the impact of specific features on classification performance.

The traditional feature extraction method has achieved good performance in ECG classification. Researchers usually fed the extracted features to the machine learning model to achieve heartbeat classification. The methods employing deep learning-based approaches have generated a competitive classification performance to the feature extraction-based methods. However, the classification performance of deep learning models can still be achieved by simple machine learning models. This means that there is still room for further performance improvements in this method.

In this paper, a heartbeat classification method based on multifeature combination and Stacking-DWKNN models is proposed to address the shortcomings of deep learning methods and traditional machine learning methods. The distance weight KNN algorithm (DWKNN) is to improve the KNN model by setting the weight of distance. The method proposed further improves the performance of the classification. The main contributions of this paper are as follows:

1. Different feature combinations are constructed. The suitability of every single feature is evaluated, and the results of different feature combinations on classification are analyzed to obtain the optimal feature combination.
2. Different model fusion methods are used for heartbeat classification to obtain the optimal model fusion method.
3. The Stacking-DWKNN model with the optimal feature combination is employed to distinguish normal beat (N), supraventricular ectopic beat (S), ventricular ectopic beat (V), and fusion normal (F), which is of great significance for clinical diagnosis.

The other parts of this paper are structured as follows.  Section 2 introduces related work. The methods of heartbeat classification are introduced in Section 3. Experimental analysis and classification results are described in Section 4.  Section 5 summarizes the full text.

## 2. Related Work

In the early days, the diagnosis of arrhythmias was based on the experience of the doctor. However, due to the diversity of arrhythmias and the corresponding complexity of the ECG waveform, manual analysis methods are no longer applicable. ECG intelligent analysis has become a research focus in recent years. Researchers have developed a diversity of classification methods for arrhythmias.

### 2.1. Arrhythmia Classification Based on Deep Learning

Deep learning does not require the manual design of feature extractors. It can automatically learn the features of ECG and extract the key features. It has very good robustness and makes the classification of heartbeat more efficient.

Some researchers [5–8] employed convolutional neural networks (CNNs), which automatically extract the ECG features and significantly improve the final prediction. Some works [9, 10] proposed a deep learning architecture based on a convolutional recurrent neural network (GRNN) to detect arrhythmias. Li et al. [11] designed the architecture of the deep neural network, CraftNet, for accurately recognizing the features, and assembled multiple child classifiers to classify heartbeats. Li et al. [12] used long short-term memory (LSTM) model to distinguish different category heartbeats. Ebrahimzadeh et al. [13] extracted a balanced combination of the Hermit features and interval features. And then, a number of multilayer perceptron (MLP) neural networks were employed to classify heartbeats.

The results of these researches were remarkable. Deep learning integrates feature learning into the process of modeling, and the classification of heartbeat is simple and effective. However, the requirement of deep learning for searching the optimal combination of features is challenging.

### 2.2. Arrhythmia Classification Based on Feature Extraction

Traditional machine learning (ML) involves direct feature engineering, making algorithms easy to interpret and understand. In addition, we have a comprehensive understanding of the algorithm and the structure of the data, making it easier to change the model. In recent years, researchers have developed numerous approaches for automatic classification. Among them, the two steps of feature extraction and classification are the most critical in the classification process, which are deeply studied by researchers. Furthermore, researches used numerous features to describe the ECG heartbeats, Hermite functions [13], morphological features [14, 15], wavelet features [16, 17], high-order statistical features [18, 19], QRS amplitude vector [20], QRS complex wave area [21], and heartbeat intervals [22–24]. Over the past few decades, numerous algorithms have been developed to distinguish different types of arrhythmias, including linear classifier [25–27], decision tree [28, 29], k-nearest neighbor [30–32], support vector machine [33, 34], random forest [35, 36], and ensemble classifier [37–41], etc.

In [27], researchers have extracted ECG morphology, heartbeat intervals, and RR-intervals and then applied a linear classifier model to the classification tasks using the learned features. Sharma et al. [32] used stop-band energy (SBE) minimized dyadic orthogonal filter bank, and wavelet decomposition of the ECG signals was performed. And then fuzzy entropy, Renyi entropy, and fractal dimension features were extracted for accurate classification. The ensemble classifiers fuse the classification results of multiple different classifiers, to achieve better performance than a single classifier. Mondéjar-Guerra et al. [34] trained specific support vector machine models for each feature, and then the multiple SVMs are combined to classify heartbeats. Shi H. et al. [37] constructed a hierarchical classifier improved by threshold and extreme gradient boosting classifier. This method has better classification performance. Javadi et al. [38] integrated a multiple neural network model based on a stacking algorithm for ECG classification, which reduced the classification error rate. Pandey et al. [39] employed an ensemble of SVMs to classify heartbeats into four classes. Rajesh et al. [40] used intrinsic mode functions to get the final features, and the AdaBoost classifier was employed to classify heartbeats. Shi et al. [41] employed a regional feature extraction method and used an ensemble classifier to distinguish heartbeats.

Although the aforementioned studies have achieved a good classification effect, the extracted medically meaningful features are less, part of the information hidden in the ECG is not easy to be revealed, the classification accuracy also needs to be improved, the classifier does not use a cross-validation method, and the robustness needs to be improved. The relevant literature in the related work is summarized in Table 1.

## 3. Methods

A typical heartbeat classification method consists of four main modules.  Figure 1 shows the frame of the classification method. The preprocessing module mainly performs denoising and segmentation. Later, 235 points near *R* peak, P length, QRS length, *T* length, PR interval, ST segment, QT interval, RR interval, *R* amplitude, and *T* amplitude are extracted from the ECG signal. Furthermore, the features are combined and normalized. Finally, the optimal feature combination is fed to the Stacking-DWKNN algorithm, and then the final classification results are obtained. In this section, each module is introduced in detail.

### 3.1. ECG Signal Preprocessing

Noise mixed in ECG signal includes baseline drift and muscle artifacts, etc. They weaken the quality of the ECG signal, make the entire ECG waveform ambiguous, and seriously affect the analysis and diagnosis of ECG signals. In this paper, to classify heartbeat more accurately, the noise of raw ECG signal is removed by wavelet transform. Wavelet transform is a signal time-frequency analysis method [42], which can retain the features of ECG signal. Besides, it avoids important physiological details and has a simple calculation process [43, 44]. The wavelet transform and wavelet basis functions are as follows:

(1) $$\begin{array}{c} W_{f}\left(m,\tau \right)=m^{-\left(1/2\right)}\int_{-\infty }^{+\infty }f\left(t\right)\psi \left(\frac{t-n}{m}\right)\text{d}t, \end{array}$$

(2) $$\begin{array}{c} \psi_{m,\tau }\left(t\right)=m^{-\left(1/2\right)}\psi \left(\frac{t-n}{m}\right),\;m>0,\tau \in R. \end{array}$$

In formula (1), *m* represents the scale factor and *n* represents the transforming parameter. They are mainly used to stretch the basic wavelet function *ψ*(*t*), *τ* reflects the displacement, and *m* and *τ* are continuous variables, so it is also called continue wavelet transform (CWT) [42].

A complete heartbeat is composed of three basic waveforms: the P, QRS, and T. The most important step in segmentation is to obtain the positions of the QRS complex. The existing R peak detection methods have obtained sufficient accuracy [45, 46]. Each heartbeat contains a pre-R segment and a post-R segment. The pre-R segment before the *R* peak contains 90 sample points, and the post-R segment after the *R* peak contains 144 sample points [47]. *R* wave is the fiducial point for waveform positioning. In this paper, the “Pan-Tompkins” algorithm is used to locate the *R* waves, and the detected *R* wave is compared with the marked *R* wave in the MIT-BIH arrhythmia database. The result of *R* wave detection is shown in Figure 2.  Table 2 shows some results of *R* wave detection in the MIT-BIH arrhythmia database.

### 3.2. Heartbeat Feature Extraction

Feature extraction is a process of extracting representative samples from a large amount of data. These samples are used as features of the final classification. According to the literature [14, 15, 20, 22–24, 29], the wavelength, interval, and morphology of ECG signals have important medical significance and can reveal the hidden information in the heartbeat. Hence, based on the detected fiducial points, the 10 feature parameters are extracted for classification in this paper.  Figure 3 is the annotation of each feature in the ECG signal.  Table 3 summarizes the features extracted in this paper and detailed as follows:

1. Single heartbeat morphology (Morph): 235 sampling points at *R* peaks from the prepared R peak annotation file are extracted as morphology features. Among them, the pre-R segment contains 90 sample points, and the pos-R segment contains 144 sample points [47]. Before the first or after last detected QRS complex reaches only 235 sampling points, then the corresponding heartbeat is used.
2. P-QRS-T: A complete ECG waveform contains P, QRS, and *T* waves. P length (P_len), QRS length (QRS_len), and *T* length (T_len) are important parameters in electrocardiogram. P-QRS-T in this paper is used to represent P, QRS, and *T* length.
3. Interval: It represents the time interval between different waveform points on the electrocardiogram. RR interval (RR_inter), QT interval (QT_inter), ST segment (ST_seg), and PR interval (PR_inter) are selected in this paper. These intervals are important for the diagnosis of arrhythmia.
4. Amplitude: *R* amplitude (R_amp) and *T* amplitude (T_amp) are selected in this paper. The *R* amplitude is the wave with the largest amplitude among all waves. The *R* amplitude is the amplitude after removing noise in this paper. The *T* wave amplitude reflects the potential changes in the later period of ventricular repolarization.

### 3.3. Feature Combination

Feature combination is to combine individual features (multiplication, splicing, or Cartesian product) to get new features. In feature combination, the first-order discrete features are often combined to form high-order combination features, so as to resolve more complex problems [48]. The morphology, interval, and amplitude of ECG signal are of great medical significance, which is very important for diagnosing arrhythmias. Because a single feature cannot fully describe the ECG signal, these three types of features are combined in stitching ways, and the effects of different feature combinations on heartbeat classification are analyzed to select the optimal combination in this paper.

### 3.4. Stacking-DWKNN Model Description

The idea of the stacking method is to use the basic classifier in the first layer to predict the training samples separately. Each DWKNN model is trained using a ten-cross-training process, which divides the training set into ten subsets. For each subset, the remaining dataset is used to train the model, and then the subsets predicted the result. This process is repeated ten times. The results are used as the training set of the secondary model and use the class label of the original data as the label of the training set of the metaclassifier. The weighted average of the ten prediction results of the test set is used for the final prediction [49].  Figure 4 presents the frame of the Stacking algorithm. And the Stacking algorithm is detailed in Table 4. The first layer of the stacking algorithm integrates four DWKNN algorithms with different parameters in this paper.

As a highly flexible and general classification algorithm, the KNN model can classify various sample distributions and has good classification ability for small sample data [50]. However, when the samples are unbalanced, it may cause that when a new sample is input, the samples of the large capacity class of the K neighbors of the sample are the majority, so the weight method can be used for improvement.

Distance-weighted k-nearest neighbor (DWKNN) is based on the KNN model. The idea of the DWKNN algorithm is to give weights to *k*-nearest neighbors according to the distances. The neighbors closer to the test sample have greater weight. A weight *w*_*i*_′ is assigned to the i-th nearest neighbor *x*_*i*_^MM^ of the test sample *x*′ in this paper; the distance-weighted is given by [50]:

(3) $$\begin{array}{c} w_{i}^{\prime }=\frac{1}{\left(\text{distance}+\text{const}\right)}. \end{array}$$

And then, the class *y*′ of the test sample *x*′ is labeled according to the majority weighted voting mechanism, and the voting formula is shown in (4) [51], where I is the indicating function, and the calculation formula of I is as follows (5) [50]:

(4) $$\begin{array}{c} y^{\prime }=\underset{y}{\arg\max}\sum_{\left(x_{i}^{\text{MM}},y_{i}^{\text{MM}}\right)\in T^{\prime }}w_{i}^{\prime }\times I\left(y=y_{i}^{\text{MM}}\right), \end{array}$$

(5) $$\begin{array}{c} I\left(y,\;y_{i}^{\text{MM}}\right)=\left\{\begin{array}{cc} 0, & y=y_{i}^{\text{MM}},\\ 1, & y\neq y_{i}^{\text{MM}}. \end{array}\right. \end{array}$$

## 4. Results

In this section, the experimental procedure is described in detail. Our focus is on feature extraction and classification. According to the medical significance of electrocardiogram, ten features are extracted, and then the effect of different feature combinations and Stacking-DWKNN algorithm on the classification results is analyzed. The MIT-BIH arrhythmia database (MIT-AD) is employed in this paper. The classification result is used as a preliminary diagnosis result of the computer to help the doctor make a further diagnosis.

### 4.1. Experimental Data

All the experiments in this paper are completed on the MIT-AD. The database consists of 48 two-lead records digitized at 360 HZ. Each of the ECG records includes one and a half hours of 2-lead dynamic ECG segments [52]. In this paper, the normal (N), supraventricular (S), ventricular (V), and fusion (F) heartbeats in MIT-AD are distinguished. The four types of heartbeats have a total of 101413 records. This paper randomly selected 90% of the heartbeat data for training and the remaining 10% for testing. The specific distribution of data is shown in Table 5.

### 4.2. Evaluation Indicator

In this paper, the data is divided into a training set and a test set, and the label output of the model is compared with the real label to get the experimental results. The results of N category heartbeat classification are calculated by formulas (6)–(9) [42]. S, V, and F heartbeats are calculated in the same way. Description of a confusion matrix is shown in Table 6, where N, S, V, and F represent the real category of heartbeat and *n*, s, *v*, and *f* represent the predicted type of heartbeat.

(6) $$\begin{array}{c} {\text{TP}}_{N}=N_{n}, \end{array}$$

(7) $$\begin{array}{c} {\text{FN}}_{N}=\text{Ns}+\text{Nv}+\text{Nf}, \end{array}$$

(8) $$\begin{array}{c} {\text{TN}}_{N}=\text{Ss}+\text{Sv}+\text{Sf}+\text{Vs}+\text{Vv}+\text{Vf}+\text{Fs}+\text{Fv}+\text{Ff}, \end{array}$$

(9) $$\begin{array}{c} {\text{FP}}_{N}=\text{Sn}+\text{Vn}+\text{Fn}. \end{array}$$

For the comprehensive evaluation of the performance, sensitivity (Se), specificity (Sp), positive predictive value (+*p*), and accuracy (Acc) are used as indicators in this paper. Higher values of these indicators indicate better classification performance. These four indicators are calculated by the following formula [42].

(10) $$\begin{array}{c} \text{Se}=\frac{\text{TP}}{\left(\text{TP}+\text{FN}\right)},\\ \text{Sp}=\frac{\text{TN}}{\left(\text{TN}+\text{FP}\right)},\\ +p=\frac{\text{TP}}{\left(\text{TP}+\text{FP}\right)},\\ \text{Acc}=\frac{\left(\text{TP}+\text{TN}\right)}{\left(\text{TP}+\text{TN}+\text{FP}+\text{FN}\right)}. \end{array}$$

### 4.3. Experiment and Result Analysis

To distinguish arrhythmia more accurately, the classification strategy using the multifeature combination and Stacking-DWKNN algorithm is proposed, which is mainly reflected in the experimental part. This section first compares and analyzes the classification results of KNN models with different feature combinations to select the optimal feature combination (Section 4.3.1); later, in order to achieve better classification results, the parameters K of the KNN model are adjusted (Section 4.3.2). Furthermore, different models are compared to verify that the KNN model is the best, and the classification results of the fusion of different models are compared to show that the framework proposed in this paper is better (Section 4.3.3), which are finally compared with other references (Section 4.3.4). Our focus is mainly on the selection of feature combinations and the influence of the model fusion method proposed in this paper on heartbeat classification.

#### 4.3.1. Analysis of Experimental Results of Different Feature Combinations

In order to select the optimal feature combination, the effects of the KNN model with different feature combinations on heartbeat classification are analyzed, and the above four indicators are used for evaluation.

15 group experiments are performed in experiment I using the KNN model with interval features. The goal of this experiment is to get the optimal interval feature combination. The classification results of the KNN model with different interval combinations are shown in Table 7. The best accuracy of 95.41% is obtained by P-QRS-T, PR_inter, QT_inter, ST_seg, and RR_inter. The optimal interval combination is represented by Inter, Inter = {P-QRS-T, QT_inter, RR_inter, PR_inter, ST_seg}.

Three groups of experiments are performed in experiment II using the KNN model with amplitude features. The goal of this experiment is to get the optimal amplitude of heartbeat classification. The classification results are represented in Table 8. Compared with the KNN model with R_amp and T_amp, using only R_amp has the same classification effect. Besides, too many heartbeat features will reduce the efficiency of the classifier, so R_amp is selected as the optimal amplitude feature.

Through the above two experiments, the best combination of interval and amplitude features is obtained. The optimal combination of the three types of features is represented by Morph, Inter, and Amp.

  Morph = {single heartbeat morphology};
  Inter = {P-QRS-T, QT_inter, RR_inter, PR_inter, ST_seg};
  Amp = {R_amp}.

In experiment III, in order to analyze the suitability of every single feature, each feature is fed into the KNN model for training. The resulting confusion matrices for the KNN model with a single feature are presented in Table 9. It is obvious that the single heartbeat morphology feature (Morph) is the best descriptor, and the number of correctly classified heartbeats is the largest.  Table 10 shows the classification results calculated from the confusion matrix. The average classification accuracy is 98.88%. From the perspective of the heartbeat, almost all the classification indicators of the KNN model with Morph features have obtained the best results, which are higher than Inter and Amp features.

In experiment IV, to compare the effect of different feature combinations on heartbeat classification, different feature combinations are fed into the KNN model. Tables 11 and 12 present confusion matrices and performance results calculated for each class. The larger the diagonal value in the confusion matrix, the better the classification effect of the classifier. It can be seen that the best results are almost based on the KNN model with Morph, Inter, and Amp features. The average classification accuracy is 98.88%. From these results, ECG information can be expressed more comprehensively by using interval, amplitude, and morphology features in heartbeat classification.

From the above experiments, it is obvious that the single heartbeat morphology is the optimal single feature for distinguishing the heartbeat. The optimal feature combination is single heartbeat morphology, Inter, and Amp features. The average classification accuracy is 98.91%.  Figure 5 shows the KNN model with optimal features combination of classification results.

#### 4.3.2. Analysis of Experimental Results with Different Parameters

To achieve better classification performance, the model parameters are adjusted. In the k-nearest-neighbor algorithm, the parameter K represents the *k* neighbors closest to the classified samples. Generally, the K value is too small, and the classification accuracy of the model is low. The K value is too large, and the model is easy to fit. To determine the appropriate K value, ten experiments are conducted with different parameters. Based on different parameter values, the classification results of the KNN model with the optimal feature combination are presented in Table 13.

It is obvious from Table 13 that when *k* = 4, the performance of the classifier is the best, with a classification accuracy of 98.91%. And the classification results of different parameters are different, indicating that the parameters have a certain influence on the classification results of the model. Afterward, the K-nearest neighbors are given different weights according to their distance from the classified samples. The accuracy of the DWKNN algorithm with the optimal feature combination is 98.96%.

#### 4.3.3. Analysis of Experimental Result Analysis of Different Classifiers

The performance of different classifiers is mainly compared in this section. From the above experiments, the optimal combination of features is Morph, Inter, and Amp. In this experiment, accuracy (Acc%) is employed as the evaluation indicator to compare the performance differences of support vector machine (SVM), random forest (RF), logistic regression (LR), linear discriminant classifier (LDA), decision tree (DT), gradient boosting decision tree (GBDT), K-nearest neighbor (KNN), and improved KNN (DWKNN) on different datasets. The classification results of the optimal feature combination based on different classifiers are presented in Table 14.

As shown in Table 14, it is obvious that the classification results of the KNN model are the best. The average classification accuracy is 98.91%. The *k*-nearest neighbors of the KNN model are given different weights (DWKNN), and the classification results are improved. The ensemble of multiple KNN models (Stacking-DWKNN) has a higher classification performance than a single model. The ensemble classifier fully utilized the correctly classified results of base learners and the difference between them. This demonstrates the outstanding performance of ensemble classifiers and does improve the results of heartbeat classification. The accuracy of the Stacking-DWKNN model with the optimal feature combination is 99.01%.

The classification result by five ensemble structures with the optimal feature combination is shown in Table 15. Table 15 lists the 16 metrics of classification results, including Se, Sp, and +*p* for each beat and the average accuracy. The Stacking-DWKNN structure has the best comprehensive classification ability: yielding the 8 highest scores on 13 metrics. It achieves the best average sensitivity and specificity of 94.26% and 98.63%. Among them, the N category and V category achieved better results. The Stacking-SVM, Stacking-DT, Stacking-GBDT, and Stacking-RF recognized the N category very well but at the cost of low detection rate of F beat. At the same time, the Stacking-DWKNN recognized the S category, and the F category is improved compared to them. This is because improving the KNN model through weights improves the impact of data imbalance.  Figure 6 shows the Stacking-DWKNN model with different features of classification results.

In order to understand the effect of different model fusion methods, based on the DWKNN (baseline1) model, different model fusion methods are used, and the optimal feature vectors are fed to different models, namely, Voting-DWKNN (baseline2), Bagging-DWKNN (baseline2), and Stacking-DWKNN (proposed) algorithm.  Table 16 shows the classification performance of different fusion methods with the optimal feature combination. The statistical measures include Se, Sp, and +*p* for each beat and the average accuracy. From these results, the Stacking-DWKNN model yields the 9 highest scores on 13 metrics; in particular, the three indicators of S-type heartbeat reached the highest, so this model is preferred for heartbeat classification.

#### 4.3.4. Comparison with Previous Studies

Table 17 shows a comparison of the classification result between the proposed method and other studies, which also perform on MIT-AD. The results show that the Stacking-DWKNN model with multiple combinations of features has better classification accuracy than the other methods discussed in this paper. And the average classification accuracy is 99.01%. The method can accurately distinguish between four categories of heartbeats. As can be seen, a comparison of the classification results from the heartbeat perspective shows that the method outperforms [8, 11, 26, 32, 34] on all metrics. Compared with [14], the positive predictive value of S beats is slightly lower, but the proposed method has obvious advantages in other indicators. Regarding the sensitivity, the method proposed in this paper achieved higher values compared to previous methods for the majority classes, N and V. But compared with the literature [33, 37], the sensitivity of class S and class F is slightly lower. This is due to the lower number of these two types of heartbeats. It can be concluded from the above that the proposed method has better classification performance. The most important arrhythmias (S and V) have all achieved better results.

## 5. Conclusions

Accurate classification of arrhythmias is essential for treating patients. Therefore, an intelligent classification method based on multifeature combination and Stacking-DWKNN algorithm is presented in this paper, which can realize the selection of ECG features and heartbeat classification. The results show that the proposed method has a good recognition rate for four heartbeats. The key points of this study are as follows:

1. Different feature combinations are constructed, and the effect of different combinations of features on heartbeat classification is evaluated to select the optimal feature combination, which provides a good application for ECG feature selection
2. The classification effects of several different classifiers are compared to select the optimal classifier, and then different model fusion methods are used for heartbeat classification based on this classifier to obtain the optimal model fusion method
3. The experimental results show that the Stacking-DWKNN model with optimal feature combination can distinguish four different types of the heartbeat

The Stacking-DWKNN model first uses DWKNN models to predict samples separately. The training process of each DWKNN model adopts a cross-training method, the prediction results are used as the input of the secondary model to make the final prediction, and then the final classification is determined by combining the classification results of multiple classifiers to achieve better performance than a single classifier. The cross-validation method effectively alleviates the overfitting problem encountered by a single classification algorithm and has strong robustness. The average classification accuracy is 99.01%.

However, the results of F-type are worse than other types because a few F-types have difficulty in analyzing the features of this type of heartbeat in detail. In the future, we need to include the use of multiple leads and add more complex feature fusion methodologies, and also more attention should be paid to improve the performance of F-type.

## Figures and Tables

**Figure 1:** The frame of heartbeat classification.

**Figure 2:** The result of R wave detection.

**Figure 3:** Annotation of heartbeat features.

**Figure 4:** Stacking algorithm structure.

**Figure 5:** Classification results of KNN model with Morph, Inter, and Amp features.

**Figure 6:** Classification result based on Stacking-DWKNN model with different feature combinations.

**Table 1:** Summary of related work.

Methods	Classifier	Literatures
Deep learning	CNN	[5–8]
	GRNN	[9, 10]
	CraftNet	[11]
	LSTM	[12]
	MLP	[13]

Machine learning	SVM	[14, 16, 20, 22, 33, 34]
	HMM	[15]
	KNN	[18, 30–32]
	SVM&ICA-PCAnet	[19]
	RF	[21, 35, 36]
	LDC	[23]
	Linear classifier	[25–27]
	DT	[28, 29]
	Ensemble	[37–41]

**Table 2:** Statistics results of *R* wave detection in MIT-BIH arrhythmia database.

Records	Fdr (%)	Se (%)	+*p* (%)	Acc (%)
100	0.04	99.96	100.00	99.96
101	0.27	100.00	99.73	99.73
103	0	100.00	100.00	100.00
106	0.59	99.56	99.85	99.41
109	0.28	100.00	99.72	99.72
113	0.06	99.94	100.00	99.94
114	0.27	99.95	99.79	99.73
117	0.07	100.00	99.93	99.93
119	0	100.00	100.00	100.00
124	0.06	99.94	100.00	99.94
202	0.38	99.62	100.00	99.62
205	0.11	99.89	100.00	99.89
208	0.82	99.53	99.66	99.18
212	0	100.00	100.00	100.00
213	0.03	99.97	100.00	99.97
215	0.03	100.00	99.97	99.97
220	0	100.00	100.00	100.00
223	0.12	99.96	99.92	99.88
228	8.19	99.90	92.51	91.81
231	0.06	99.94	100.00	99.94
232	0.79	100.00	99.22	99.21
234	0.07	99.93	100.00	99.93
**Total avg**	**0.56**	**99.91**	**99.56**	**99.44**

*Note.* The first column is the record name, the second column is the evaluation indicator “false detection rate,” the third column is the evaluation indicator “sensitivity,” the fourth column is the evaluation indicator “positive predictive value,” and the fifth column is the evaluation indicator “accuracy.” According to the AAMIEC38 standard, the difference between the detected QRS complex and the manual mark is within 150 ms, which means that the location detection is successful.

**Table 3:** Ten values of ECG signal features in this paper.

Number	ECG signal features	Introduction of ECG signal feature parameters
1	Morph	235 points of a single heartbeat
2	P_len	The time between the start and end of the P wave
3	QRS_len	The time between the start and end of the QRS complex
4	T_len	The time between the start and end of the *T* wave
5	RR_inter	The time between two adjacent *R* waves
6	PR_inter	The time from the start of the P wave to the start of the QRS complex
7	ST_seg	The time from the end of the QRS wave to the start of the *T* wave
8	QT_inter	The time between the QRS wave and the *T* wave
9	R_amp	The maximal of the *R* wave
10	T_amp	The maximal of the *T* wave

**Table 4:** The description of Stacking-DWKNN algorithm.

Algorithm 1: Stacking-DWKNN algorithm

**Input:** dataset *D*={(*x*_1,_*y*_1_), (*x*_2,_*y*_2_), ..., (*x*_*t*,_*y*_*t*_)}
**Output:** ensemble classifier H (DWKNN model)
1: learn the base classifiers
2: **for ***s* = 1 to S **do**
3: learn *h*_*s*_(DWKNN model) based on D
4: **end for**
5: Generate a new dataset for prediction
6: **for ***i* = 1 to *t ***do**
7: *D*_*h*_={*x*_*i*_′, *y*_*i*_}, where *x*_*i*_′={*h*_*i*_(*x*_*i*_), ..., *h*_*s*_(*x*_*i*_)}
8: **end for**
9: learn a metaclassifier
10: learn H based on *D*_*s*_
11: return H

**Table 5:** Experimental data statistics.

	Training set	Testing set	Total
**N**	81,560	9,035	90,595
**S**	2,528	253	2,781
**V**	6,450	785	7,235
**F**	723	79	802

**Table 6:** Confusion matrix of classification results.

	n	s	v	f	Total
**N**	Nn	Ns	Nv	Nf	∑*N*
**S**	Sn	Ss	Sv	Sf	∑*S*
**V**	Vn	Vs	Vv	Vf	∑*V*
**F**	Fn	Fs	Fv	Ff	∑*F*

**Table 7:** Classification results of the KNN model with interval features.

Features					Evaluation metrics (%)
P-QRS-T	RR_inter	PR_inter	ST_seg	QT_inter	Acc
•	•				92.17
•		•			90.89
•			•		92.85
•				•	91.78
•	•	•			92.72
•	•		•		94.71
•	•			•	94.68
•		•	•		93.92
•		•		•	93.10
•			•	•	94.53
•	•	•	•		95.39
•	•	•			95.27
•	•		•	•	94.76
•		•	•	•	95.26
•	•	•	•	•	**95.41**

**Table 8:** Classification results for the KNN model with amplitude features.

Features		Evaluation metrics (%)
T_amp	R_amp	Acc
•		89.42
	•	**90.26**
•	•	90.26

**Table 9:** Confusion matrix for the KNN model combining with single features.

	Morph				Inter				Amp			
	n	s	v	f	n	s	v	f	n	s	v	f
N	9009	12	12	2	8939	26	56	14	8960	20	53	2
S	40	271	1	0	135	169	8	0	306	6	0	0
V	23	0	690	3	162	5	544	5	527	3	186	0
F	12	1	8	57	47	0	7	24	68	0	9	1

**Table 10:** Confusion matrix for the KNN model combining with single features.

	Morph				Inter				Amp			
	Se(%)	Sp(%)	+*p*(%)	Acc(%)	Se(%)	Sp(%)	+*p*(%)	Acc(%)	Se(%)	Sp(%)	+*p*(%)	Acc(%)
N	**99.71**	**93.22**	**99.17**	**99.00**	98.94	68.90	96.29	95.66	99.17	18.54	90.86	90.38
S	**86.86**	**99.87**	**95.42**	**99.47**	54.17	99.68	84.50	98.28	19.20	99.77	20.69	96.76
V	**96.37**	**99.78**	**97.05**	**99.54**	75.98	99.25	88.46	97.60	25.98	99.34	75.00	94.16
F	**73.08**	99.95	**91.94**	**99.74**	30.77	99.81	55.81	99.28	12.80	99.98	33.33	99.22

**Table 11:** Confusion matrix for the KNN model combining with different feature combinations.

	Morph + Inter				Morph + Amp				Inter + Amp				Morph + Inter + Amp			
	N	s	v	f	n	s	v	f	n	s	v	f	n	s	v	f
N	9010	12	11	2	9010	12	11	2	8942	27	54	12	9009	13	11	2
S	42	269	1	0	40	271	1	0	77	224	11	0	37	274	1	0
V	22	2	691	1	23	0	690	3	85	8	619	4	22	2	691	1
F	15	0	7	56	12	1	8	57	28	0	9	41	15	0	7	56

**Table 12:** Classification performance for KNN model trained with different feature combinations.

	Morph + Inter				Morph + Amp				Inter + Amp				Morph + Inter + Amp			
	Se%	Sp%	+*p*%	Acc%	Se%	Sp%	+*p*%	Acc%	Se%	Sp%	+*p*%	Acc%	Se%	Sp%	+*p*%	Acc%
N	**99.72**	92.86	99.13	98.97	**99.72**	93.22	99.17	**99.01**	98.97	82.82	97.92	97.21	99.71	**93.31**	**99.19**	**99.01**
S	86.22	99.86	95.05	99.44	86.86	**99.87**	**95.42**	99.47	71.79	99.64	86.49	98.79	**87.82**	99.85	94.81	**99.48**
V	**96.51**	99.79	**97.32**	**99.57**	96.37	99.79	97.18	99.55	86.45	99.21	89.32	98.31	**96.51**	**99.80**	**97.32**	**99.57**
F	**71.79**	**99.97**	**94.92**	**99.76**	73.08	99.95	91.94	99.74	52.56	99.84	71.93	99.48	**71.79**	**99.97**	**94.92**	**99.75**

**Table 13:** Classification results of different K values.

Parameter K	1	2	3	4	5	6	7	8	9	10
Acc (%)	98.84	98.80	98.85	**98.91**	98.79	98.80	98.72	98.74	98.65	98.65

**Table 14:** Classification results of different classifiers trained with all possible feature combinations.

Feature combination			Classifier								
Morph	Inter	Amp	LDA	LR	SVM	DT	GBDT	RF	KNN	DW KNN	Stacking-DWKNN
•			91.71	92.39	98.61	97.35	97.61	98.55	98.88	98.95	**98.94**
	•		89.06	89.01	93.69	93.47	94.45	95.73	95.41	95.36	**95.59**
		•	90.42	89.14	90.59	87.98	90.58	87.81	90.26	88.47	**90.43**
•	•		93.03	93.25	98.69	97.43	97.73	98.57	98.87	98.97	**98.97**
•		•	91.74	92.40	98.69	97.47	97.55	98.58	98.89	98.94	**98.95**
	•	•	90.14	90.94	95.71	95.74	96.01	97.08	96.89	96.93	**97.09**
•	•	•	93.82	94.24	98.74	97.80	98.15	98.83	98.91	98.96	**99.01**

**Table 15:** Classification performance for stacking model combined with different classifier combinations.

	N			S			V			F			Acc
	Se(%)	Sp(%)	+*p*(%)	Se(%)	Sp(%)	+*p*(%)	Se(%)	Sp(%)	+*p*(%)	Se(%)	Sp(%)	+*p*(%)	Num
Stacking-SVM	99.83	91.32	98.95	81.09	99.96	98.44	96.51	**99.78**	97.05	69.32	**99.98**	**96.43**	98.79
Stacking-DT	98.93	90.96	98.89	81.73	99.50	83.88	93.99	99.51	93.60	70.51	99.75	68.75	97.83
Stacking-GBDT	99.68	88.16	98.57	74.68	99.90	95.88	94.41	99.71	96.16	66.67	99.94	89.66	98.28
Stacking-RF	**99.86**	91.68	98.99	82.05	**99.98**	**99.22**	96.51	**99.78**	97.05	70.51	**99.98**	96.49	98.85
Stacking-DWKNN	99.65	**94.94**	**99.38**	**89.42**	99.85	94.90	**97.21**	**99.78**	**97.07**	**80.77**	99.94	88.73	**99.01**

**Table 16:** Classification performance of fusion of different models.

	N			S			V			F			Avg
	Se(%)	Sp(%)	+*p*(%)	Se(%)	Sp(%)	+*p*(%)	Se(%)	Sp(%)	+*p*(%)	Se(%)	Sp(%)	+*p*(%)	Acc (%)
Baseline1	99.60	94.85	99.37	88.78	99.79	92.95	97.20	99.80	97.35	80.77	99.92	88.73	98.96
Baseline2	99.58	92.86	99.13	87.18	99.77	92.20	95.95	99.76	96.76	70.51	99.94	**91.67**	97.83
Baseline3	**99.67**	94.39	99.32	89.10	99.81	93.60	96.51	**99.81**	**97.46**	78.21	99.93	89.71	98.95
Proposed	99.65	**94.94**	**99.38**	**89.42**	**99.85**	**94.90**	**97.21**	99.78	97.07	**80.77**	**99.94**	88.73	**99.01**

**Table 17:** Comparison with other studies.

Reference	Features	Classifier	Performance
Mar et al. [26]	Statistical features + SFFS; temporal features; morphological features	Weighted LD, MLP	Acc = 89.9%;
			Se_n_ = 89.6%; +*P*_n_ = 99.1%:
			Se_s_ = 83.2%; +*P*_s_ = 33.5%;
			Se_v_ = 86.8%; +*P*_v_ = 75.9%;
			Se_f_ = 61.1%; +*P*_f_ = 16.6%;

Zhang et al. [33]	ECG-intervals and segments; RR interval; morphological features	Combined SVM	Acc = 86.66%;
			Se_n_ = 88.94%; +*P*_n_ = 98.98%:
			Se_s_ = 79.06%; +*P*_s_ = 35.98%;
			Se_v_ = 85.48%; +*P*_v_ = 92.75%;
			Se_f_ = 93.81%; +*P*_f_ = 13.73%;

Zhu et al. [14]	ECG morphology	SVM	Acc = 97.80%;
			Se_n_ = 99.27%; +*P*_n_ = 98.48%;
			Se_s_ = 87.47%; +*P*_s_ = 95.25%;
			Se_v_ = 94.71%; +*P*_v_ = 95.22%
			Se_f_ = 73.88%; +*P*_f_ = 86.09%

Mondéjar-Guerra [34]	RR interval; HOS; ECG morphology; wavelet coefficients	Ensemble SVM	Acc = 94.5%;
			Se_n_ = 95.9%; +*P*_n_ = 98.2%;
			Se_s_ = 78.1%; +*P*_s_ = 49.7%;
			Se_v_ = 94.7%; +*P*_v_ = 93.9%
			Se_f_ = 12.4%; +*P*_f_ = 23.6%

Shi et al. [37]	ECG morphology	Hierarchical classifier	Se_n_ = 92.1%; +*P*_n_ = 99.5%;
			Se_s_ = 91.7%; +*P*_s_ = 46.2%;
			Se_v_ = 95.1%; +*P*_v_ = 88.1%;
			Se_f_ = 61.6%; +*P*_f_ = 15.2%;

Sharma et al. [32]	Fuzzy entropy; Renyi entropy; fractal dimension	KNN	Acc = 94.5%;
			Se_n_ = 99.59%; Sp_n_ = 91.92%; +*P*_n_ = 98.34;
			Se_s_ = 73.64%; Sp_s_ = 99.84%; +*P*_s_ = 92.09;
			Se_v_ = 92.11%; Sp_v_ = 99.75%; +*P*_v_ = 96.37;
			Se_f_ = 64.46%; Sp_f_ = 99.94%; +*P*_f_ = 88.38;

Singh et al. [8]	Gabor; wave; interval	DCNN	Acc = 93.19%;
			Se = 93.98%;
			Sp = 95%;

Li et al. [11]	R-R intervals; wavelet transform; Morph; higher-order statistics	CraftNet	Acc = 89.24%;
			Se_n_ = 88.16%; Sp_n_ = 94.34%
			Se_s_ = 85.37%; Sp_s_ = 94.85%
			Se_v_ = 94.53%; Sp_v_ = 99.70%
			Se_f_ = 88.92%; Sp_f_ = 94.28%

Proposed	Intervals; P-QRS-T wave; amplitude; ECG morphology	Stacking-DWKNN	Acc = 99.01%;
			Se_n_ = 99.65%; Sp_n_ = 94.94%; +*P*_n_ = 99.38;
			Se_s_ = 89.42%; Sp_s_ = 99.85%; +*P*_s_ = 94.90;
			Se_v_ = 97.21%; Sp_v_ = 99.78%; +*P*_v_ = 97.07;
			Se_f_ = 80.77%; Sp_f_ = 99.94%; +*P*_f_ = 88.73;

## Data Availability

(1) All datasets used to support the findings of this study are included within the article. (2) All datasets used to support the findings of this study were supplied by the publicly available MIT-BIH database from the Massachusetts Institute of Technology. The URL to access this data is https://www.physionet.org/cgi-bin/atm/ATM. (3) The coding used to support the findings of this study has not been made available because the source code in this article is part of a national project and is a trade secret, so the source code is not available.
